The article "Adolescents' Contraceptive Uptake in Ethiopia: A Meta-Analysis" was published in 2022. Journal: Biomed Res Int.

# Adolescents' Contraceptive Uptake in Ethiopia: A Meta-Analysis

**DOI:** 10.1155/2022/6104467

**Published:** 2022-08-16

**Authors:** Alemayehu Gonie Mekonnen, Daniel Bogale Odo, Dabere Nigatu

**Affiliations:** ^1^School of Nursing and Midwifery, Asrat Woldeyes, Health Science Campus, Debre Berhan University, Debre Berhan, Ethiopia; ^2^School of Public Health, College of Health Sciences, Arsi University, Asela, Ethiopia; ^3^School of Public Health, College of Medicine and Health Sciences, Bahir Dar University, Bahir Dar, Ethiopia

## Abstract

**Introduction:**

Ethiopia has made significant efforts to enhance family planning services despite variations in the community's use of modern contraception in different parts of the country. Various studies have reported the proportion and determinant factors of adolescents' contraceptive uptake in Ethiopia. These studies are not consistent in terms of size, scope, and geographic coverage, and the results need to be systematically collated to inform policies. Therefore, this review was aimed at analyzing the findings of those primary studies to obtain more representative evidence of adolescents' contraceptive uptake in Ethiopia.

**Methods:**

Five databases (MEDLINE via PubMed, Google Scholar, Scopus, ScienceDirect, and CINAHL) were searched for papers published from January 2000 up to June 2022 in English. Of thirty eligible studies, eight papers were included in this meta-analysis. Between-study heterogeneity was evaluated by the forest plot and inconsistency index (*I*^2^). A random-effects model was used to calculate the pooled estimates of adolescents' contraceptive uptake.

**Results:**

The overall pooled proportion of adolescents' contraceptive uptake was 40% (*I*^2^ = 99.70, *p* ≤ 0.001; 95%CI = 19, 61). Adolescents' usage of contraception was influenced by a number of factors: individual-, sociocultural-, knowledge- (about contraceptive methods), and healthcare service-related factors. Individual-related factors include the educational status of adolescents, being of young age, and the income status of adolescents' families. Sociocultural-related factors comprise discussion with the family/relatives, parent disapproval and pressure from partners, and being married or having a partner. Healthcare service-related factors include the availability of youth clubs and inconvenient service hours for SRH services. Knowing contraceptive methods and SRH services was also positively associated with adolescents' contraceptive utilization.

**Conclusions:**

The proportion of adolescents who used contraception in Ethiopia was 40%. Adolescents' use of contraceptives was influenced by a variety of factors: individual-, sociocultural-, healthcare-, and knowledge-related factors. Hence, integrated interventions targeted at tackling barriers to contraceptive uptake may be helpful to improve adolescents' contraceptive utilization in Ethiopia.

The article "Adolescents' Contraceptive Uptake in Ethiopia: A Meta-Analysis" was published in 2022. Journal: Biomed Res Int.

## 1. Introduction

According to the World Health Organization (WHO) definition, adolescents are those who fall within the age range of 10 to 19 years old [1]. Adolescence is a period when people are transitioning from childhood to adulthood, and it is marked by major physical and psychological changes [1, 2]. During this period, adolescents are sexually active and have special sexual and reproductive health (SRH) needs [1, 3]. As a result of this, around 16 million adolescents give birth every year worldwide, of which greater than ninety percent of deliveries occur in low-income countries including Ethiopia [4].

The available studies indicated that female adolescents had a higher risk of dying from pregnancy-related complications as compared to adult women because their reproductive organs are not fully matured and they are not also taking contraceptive methods to prevent unwanted pregnancies [2, 5]. Additionally, anticipated stigmas resulting from societal norms and beliefs about contraceptive methods such as fear of being seen by others and embarrassment in seeking contraceptive methods [6] were the major barriers that influence adolescents from utilizing contraceptives [7]. It has been observed that many adolescents engage in unsafe sex that can result in an unwanted pregnancy, which could end up in unsafe abortion or teenage childbearing, which further constitutes the leading cause of preventable adolescent mortality and morbidity [8, 9].

At both the societal and personal levels, adolescent pregnancies and being unable to make an informed decision about their pregnancy have distinct and detrimental effects [9]. They frequently lack the social and financial resources to care for their newborns, which may be a factor in their decision to drop out of school [10, 11]. When adolescents have restricted access to contraception, their well-being and autonomy could also be compromised [12]. Additionally, the health of the newborn in adolescent women is at risk for preterm birth, low birth weight, and neonatal mortality [12–14].

Ethiopia has made significant efforts in family planning programs for the past 20 years, despite the use of modern family planning methods that vary in different parts of the community [14]. Contraceptives are available free of charge in all health facilities in the country [15]. Positive growth was seen in the national modern contraceptive prevalence rate, which rose from 8% in 2000 to 36% in 2016 [16]. Nevertheless, this achievement is still below the global FP target as adolescents, the largest segment of the population in Ethiopia, are left out of FP intervention programs and many adolescents' contraceptive needs are generally not taken into account [17, 18]. Besides, the linkage between primary healthcare facilities and households has not been strong enough to deliver ideal contraceptive services for the majority of adolescents [19–21].

The article "Adolescents' Contraceptive Uptake in Ethiopia: A Meta-Analysis" was published in 2022. Journal: Biomed Res Int.

Various studies have reported the proportion and determinant factors of adolescents' contraceptive uptake in different parts of the country [12, 20–26]. However, these primary studies are not consistent in terms of size, scope, and geographic coverage. Additionally, varying results were stated across individual studies and the results need to be systematically collated so that simple, practical, and applicable policies can be made. Therefore, this review was aimed at analyzing the findings of primary studies to obtain more representative evidence of adolescents' contraceptive uptake in Ethiopia.

## 2. Main Text

### 2.1. Search Strategy

The researchers used the Preferred Reporting Items for Systematic Reviews and Meta-Analyses (PRISMA) [27] to answer two research questions: “what is the overall proportion of adolescents' contraceptive uptake in Ethiopia?” and “what are the determinants of adolescents' contraceptive uptake in Ethiopia?” Five databases (MEDLINE via PubMed, Google Scholar, Scopus, ScienceDirect, and CINAHL) were searched for papers published from January 2000 up to June 2022 in English. The researchers limited their search to start in January 2000 since the health of adolescents has been given more attention after this period and there were not many studies on adolescents in the literature before the 2000s.

The following search terms were employed to look for articles from the abovementioned databases: social *OR* cultural *AND* determinants *OR* factors *OR* barriers *AND* adolescents *OR* teenage *AND* family planning *OR* contraceptive *AND* uptake *OR* utilization *OR* use *AND* Ethiopia. As indicated above, alternative keywords were combined using the Boolean operator “*OR*” to ensure all possible variations were captured; the search has then combined with “*AND*” to narrow the search. The following limits were applied: English, full text available online, and published between January 2000 and June 2022.

### 2.2. Inclusion and Exclusion Criteria

For papers to be included in the analyses, they had to meet the following requirements: they had to be primary cross-sectional, cohort, or mixed-method studies that were focused on family planning or contraception and were conducted in Ethiopia among adolescents and youths aged 10 to 19 years. They also had to have been published in English between January 2000 and June 2022 and have their full texts available online. A paper was excluded if it was a systematic review and included anyone beyond the age of 19 years.

The article "Adolescents' Contraceptive Uptake in Ethiopia: A Meta-Analysis" was published in 2022. Journal: Biomed Res Int.

### 2.3. Data Extraction

Two researchers (AGM and DN) independently searched and screened the titles and abstracts against the inclusion/exclusion criteria. Articles found suitable by titles and abstracts underwent full-text review. All of the retrieved full texts were reviewed by the three authors (AGM, DN, and DBO), and the data was then extracted into a summary table. Authors, year of publication, study design and setting, and characteristics of participants (study population and sample size) were extracted. The researchers also collected data on the proportion of contraceptive uptake and the key determinant variables that influence adolescents' contraceptive use (Table 1).

### 2.4. Quality Appraisal of the Included Studies

The researchers used the Newcastle-Ottawa Scale (the most widely used guideline for reporting observational studies) [28] and the Mixed Methods Appraisal Tool for quality assessment of the selected studies [29]. Each element of quality assessment was labeled as follows: 1 = a criterion was met and 0 = a criterion was not met. A study was considered a very good study when the sum of the criteria is within 9-10, a good study when the sum of the criteria is within 7-8, and satisfactory when the sum of the criteria is within 5-6 scores. All the included studies scored above 7, and they are included in the meta-analysis.

## 3. Results

### 3.1. Characteristics of Included Studies

Figure 1 shows a flowchart of the search and results. The initial search yielded 265 records, and 43 duplicates were removed. Overall, 191 papers were removed after the screening of titles and abstracts against the inclusion/exclusion criteria. Of the 31 papers remaining, 30 were retrieved in full text and assessed against the inclusion/exclusion criteria; the full text of one paper was not found. Another 22 papers were excluded in this step. To find any more papers that may not have been found in the original search, the reference lists of the included papers were scanned: 1 paper was included. Finally, 8 papers met the inclusion criteria and made eligible studies for the final analysis [12, 20–26]. Of 8 included papers, seven studies were quantitative and one study was a mixed-method approach [26] (Figure 1).

### 3.2. Sensitivity Analysis

Sensitivity analysis was done to test whether a particular study was responsible for the presence of high heterogeneity. The results confirm no statistical source of heterogeneity among the included studies in which the estimated points of each study are within the confidence interval of the pooled estimate (Figure 2).

The article "Adolescents' Contraceptive Uptake in Ethiopia: A Meta-Analysis" was published in 2022. Journal: Biomed Res Int.

### 3.3. Heterogeneity Test

Between-study heterogeneity was evaluated by the forest plot and inconsistency index (*I*^2^). The included studies were assessed for heterogeneity using the random-effects model. The random-effects model minimizes the occurrence of heterogeneity of various included studies than the fixed-effects model [29]. There was considerable heterogeneity among studies, and the true variability among the included studies other than chance was 99.7% (*I*^2^ = 99.7%) (Figure 3).

### 3.4. The Pooled Estimates of Adolescents' Contraceptive Uptake

The first aim of this analysis was to estimate the pooled proportion of adolescents' contraceptive use by using proportions measured in primary studies. Eight studies were assessed to estimate the pooled proportion of adolescents' contraceptive uptake, and the estimated points of each study are within the confidence interval of the pooled estimate. The proportion of adolescents' contraceptive uptake ranged from 12% (95%CI = 11, 14) [26] to 79% (95%CI = 77, 82) [12]. The overall pooled proportion of adolescents' contraceptive uptake was 40% (*I*^2^ = 99.70, *p* ≤ 0.001; 95%CI = 19, 61). The pooled proportion is presented in a forest plot (Figure 3).

### 3.5. Factors of Adolescents' Contraceptive Uptake

Based on their similarities, the researchers categorized the factors that influence adolescents' use of contraceptives into four thematic summaries: individual-, sociocultural-, knowledge- (about contraceptive methods), and healthcare service-related factors.

From eight studies that examined the determinants of adolescents' contraceptive uptake, the educational status of adolescents was the main factor influencing the uptake of contraceptives, and this is reported in four studies [12, 20, 24, 26]. Being of young age [22, 26] and the income status of adolescents' families [24] were significantly associated with contraceptive utilization. Sociocultural-related factors are the most commonly stated determinants of adolescents' contraceptive uptake and are mentioned in five studies [12, 21–24]. Discussion with the family/relatives and parents [12, 21], parent disapproval and pressure from partners [22], and being married or having a partner [26] were reported as the most important determinants for adolescents' contraceptive uptake.

Healthcare service-related reasons that influence the uptake of contraceptives by adolescents were raised in four studies [21, 22, 24, 25]. Availability of youth clubs and SRH services [21, 22], inconvenient service hours for SRH, and lack of information about FP [24, 25] were negatively associated with adolescents' contraceptive utilization. Having knowledge of contraceptive methods [23] and basic knowledge of SRH [21] and being informed about contraceptives through media [26] were knowledge-related determinants of adolescents' contraceptive uptake that were mentioned in three studies and found to be positively associated with adolescents' contraceptive utilization.

The article "Adolescents' Contraceptive Uptake in Ethiopia: A Meta-Analysis" was published in 2022. Journal: Biomed Res Int.

## 4. Discussions

In this meta-analysis, the researchers estimated the pooled proportion of adolescents' contraceptive utilization and thoroughly reviewed the factors that influence their contraceptive uptake in Ethiopia, where adolescents' contraceptive use remains very low [30, 31]. Summarizing the factors that influence adolescents' contraceptive use is critical to improving the well-being of the adolescent population, a population segment that is often underrepresented in the majority of modern contraception studies [30, 32]. The results in this analysis are based on eight primary studies that had been published within the last twenty years.

Overall, the pooled proportion of adolescents' contraceptive uptake was 40% in Ethiopia. A mixed-effects multilevel analysis of data from 29 demographic and health surveys in sub-Saharan Africa revealed that only 24.7% of adolescents used modern contraceptive methods, which is consistent with our findings [31]. Li et al. in their review also reported that 31.6% of female adolescents utilized modern contraceptives [33]. This shows that the proportion of adolescents' contraceptive uptake still remains very low and needs integrated work to avoid unwanted adolescent pregnancies and associated complications. Preventing unwanted pregnancies could be not only beneficial for adolescents but also helpful for their newborns and society at large [34].

In this review, individual factors such as the educational status of adolescents [12, 20, 24, 26], being of young age [22, 26], and the income status of adolescents' families [24] were associated with adolescents' contraceptive utilization. Those completing high school and belonging to the highest wealth quintile families have more access to modern contraceptive information that can promote contraceptive use [14, 33]. Evidence suggested that having a good education and being from a wealthy family can contribute to the probable improvement of contraceptive uptake by reducing gender inequality and promoting discussion with their partners or relatives, which in turn increase their utilization of contraceptive methods [13, 35]. It is also important to note that adolescents who are educated and supported financially by their families are less likely to be influenced by peers and more likely to have the freedom to decide their fertility independently [23]. On the other hand, being in a lower grade and being of young age can discourage contraceptive use as those adolescents have limited sources of information and access to contraceptive services.

The article "Adolescents' Contraceptive Uptake in Ethiopia: A Meta-Analysis" was published in 2022. Journal: Biomed Res Int.

In this review, discussion with the family/relatives and parents [12, 21], parent disapproval and pressure from partners [22], and being married or having a partner [26] were reported as the key factors influencing adolescents' contraceptive uptake. In Mali [36], Kenya [37], Ghana [11], and other low- and middle-income countries [31], the influences of social norms regarding sexual activity such as negative beliefs about contraceptive methods and feeling embarrassment at seeking contraceptive methods were reported as the major determinants of adolescents' contraceptive uptake. Barriers to adolescents' contraceptive uptake are not only restricted at the community level; they also exist among healthcare providers. For example, disapproving attitudes such as judgmental behavior and unfriendly service provision, which could have a negative impact on contraceptive service use by adolescents, were reported in previous studies in Nigeria and Tanzania [14, 30].

Healthcare service-related reasons that influence the uptake of contraceptives were raised in four studies [21, 22, 24, 25]. These include the availability of youth clubs and SRH services [21, 22], inconvenient service hours for SRH, and lack of information about FP [24, 25]. This result was comparable with findings elsewhere in Africa [3, 10, 36]. This indicates that creating a welcoming environment at health facilities and enhancing the quality of family planning services provided to adolescents could play an important role in the initiation and the continuation of contraceptive method use [37].

Having knowledge of contraceptive methods [23] and basic knowledge of SRH [21] and being informed about contraceptives through media [26] were knowledge-related factors of adolescents' contraceptive uptake that were mentioned in three studies and found to be positively associated with adolescents' contraceptive use. The role of knowledge of SRH services including contraceptive methods in our review was supported by earlier findings [5, 34]. This may show how adolescents' understanding of contraceptive methods might result in positive behavioral changes that improve their demand to utilize contraception. It is important to make adolescents more informed about contraceptive methods and other health risks they may face while pregnant.

### 4.1. Limitations of the Study

This meta-analysis may have some limitations. All of the included primary studies were cross-sectional and mixed-method studies and are more likely to be affected by the risk of reporting bias. This study is based only on published studies, and important data might be missed from unpublished studies.

The article "Adolescents' Contraceptive Uptake in Ethiopia: A Meta-Analysis" was published in 2022. Journal: Biomed Res Int.

## 5. Conclusions

In Ethiopia, the total proportion of adolescents who used contraception was low. Adolescents' use of contraceptives was influenced by a variety of factors: individual-, sociocultural-, healthcare-, and knowledge-related factors. Hence, integrated interventions targeted at overcoming barriers to contraceptive uptake may be helpful to improve adolescents' contraceptive utilization in Ethiopia.

## Figures and Tables

**Figure 1:** PRISMA diagram of the search process, June 2022.

**Figure 2:** Sensitivity analysis showing heterogeneity among the included studies, June 2022.

**Figure 3:** Forest plot of the proportion of adolescents' contraceptive uptake in Ethiopia, June 2022.

**Table 1:** Characteristics of the included studies, June 2022.

Author	Study design	Study setting	Study population	Sample size	Uptake of FP	Reported factors influencing the uptake of contraceptives
Feleke et al. [12]	Cross-sectional	Gondar town	Both male and female	1290	79.5%	Educational status of adolescents, discussion with the family/relatives, and sexual partners were associated with FP utilization
Teshome et al. [20]	Cross-sectional	Pathfinder database	Both male and female	973	66.3	Educational status and discussion with health extension workers were associated with contraceptive use
Habte et al. [21]	Cross-sectional	Southern Ethiopia	Both male and female	366	23.8	Availability of youth clubs, participation in peer education, discussion with parents, and lack of knowledge on SRH were associated with contraceptive use
Abajobir and Seme [22]	Cross-sectional	Machakel district	Both male and female	415	21.5	Being of young age, lack of basic knowledge of SRH, parent disapproval, and peer pressure discouraged adolescents from FP use
Hidata et al. [23]	Cross-sectional	Toke Kutaye district	Both male and female	1076	40.3	Discussion with friends and knowing FP methods were factors of contraceptive use
Olika et al. [24]	Cross-sectional	National survey	Female	504	39.6%	Income status of adolescents' families, educational status, and information about FP were associated with FP use
Ansha et al. [25]	Cross-sectional	Anchar district	Both male and female	402	39.3%	Lack of SRH services, lack of privacy and inconvenient service hours, and religious opposition influence adolescents' FP use
Abebe et al. [26]	Cross-sectional	Tigray region	Female	1755	12.3	Being of young age, educational status, being married/having a partner, and being informed of FP through media were factors for FP use

The article "Adolescents' Contraceptive Uptake in Ethiopia: A Meta-Analysis" was published in 2022. Journal: Biomed Res Int.

## Data Availability

All data generated/analyzed during this study are included in this published article. Besides, the row datasets will be available from the corresponding author on a reasonable request.

## Abbreviations

AOR: Adjusted odds ratio
CI: Confidence interval
FP: Family planning
NA: Not applicable
SRH: Sexual and reproductive health
PRISMA: Preferred Reporting Items for Systematic Reviews and Meta-Analyses
WHO: World Health Organization.
